The article "Clinical Efficacy of Mechanical Traction as Physical Therapy for Lumbar Disc Herniation: A Meta-Analysis" was published in 2022. Journal: Comput Math Methods Med.

# Clinical Efficacy of Mechanical Traction as Physical Therapy for Lumbar Disc Herniation: A Meta-Analysis

**DOI:** 10.1155/2022/5670303

**Published:** 2022-06-21

**Authors:** Wenxian Wang, Feibing Long, Xinshun Wu, Shanhuan Li, Ji Lin

**Affiliations:** ^1^Department of Spinal Surgery, The First Affiliated Hospital of Hainan Medical University, Haikou, 570102 Hainan, China; ^2^Department of Surgery, Hainan Cancer Hospital, Haikou, 570100 Hainan, China; ^3^Department of Orthopedics, Wenchang City People's Hospital, Wenchang, 571300 Hainan, China

## Abstract

**Objective:**

This study is aimed at exploring the clinical effect of mechanical traction on lumbar disc herniation (LDH).

**Methods:**

Related literatures were retrieved from PubMed, Medline, Embase, CENTRAL, and CNKI databases. Inclusion of literature topic was comparison of mechanical traction and conventional physical therapy for lumbar disc herniation. Jadad scale was used to evaluate the quality of the included RCT studies. The Chi-square test was used for the heterogeneity test, and a random effect model was used with heterogeneity. Subgroup analysis and sensitivity analysis were used to explore the causes of heterogeneity. If there was no heterogeneity, the fixed effect model was used, and funnel plots were used to test publication bias.

**Results:**

Visual analog scale (VAS) in the mechanical traction group was lower than that in the conventional physical therapy group (MD = −1.39 (95% CI (-1.81, -0.98)), *Z* = 6.56, and *P* < 0.00001). There was no heterogeneity among studies (Chi^2^ = 6.62, *P* = 0.25, and *I*^2^ = 24%) and no publication bias. Oswestry disability index (ODI) in the mechanical traction group was lower than that in the conventional physical therapy group (MD = −6.34 (95% CI (-10.28, -2.39)), *Z* = 3.15, and *P* = 0.002). There was no heterogeneity between studies (Chi^2^ = 6.27, *P* = 0.18, and *I*^2^ = 36%) and no publication bias. There was no significant difference in Schober test scores between the mechanical traction group and the conventional physical therapy group (MD = −0.40 (95% CI (-1.07, 0.28)), *Z* = 1.16, and *P* = 0.25). There was no heterogeneity among studies (Chi^2^ = 1.61, *P* = 0.66, and *I*^2^ = 0%) and no publication bias.

**Conclusion:**

Mechanical traction can effectively relieve lumbar and leg pain and improve ODI in patients with lumbar disc herniation but has no significant effect on spinal motion. The therapeutic effect of mechanical traction was significantly better than that of conventional physical therapy. Lumbar traction can be used in conjunction with other traditional physical therapy.

## 1. Introduction

Lumbar disc herniation (LDH), as the most common cause of low back and leg pain [1], was diagnosed in 60% to 80% of people at different ages [2]. The LDH is common in people aged 25 to 55 spending large percent of times sitting or standing with heavy workload. Current clinical treatment of LDH includes surgical treatment and nonsurgical treatment [3, 4]. Although the effect of surgical treatment is good, it faces the risk of nerve injury and adjacent vertebral bodies and recurrence [5]. Most patients with LDH are most likely treated conservatively [3, 6, 7]. Conservative treatment takes physical therapy as the primary treatment method, including hot compress, acupuncture, massage, bed rest, electrotherapy, and traction [8–10].

Lumbar traction has been widely used in the clinic; however, its clinical effect has been controversial. Lumbar traction is limited in eliminating the physical and mechanical compression of nerve roots in a short time [11] and will increase the risk of lumbar injury [12]. The known side effect of lumbar tract is pain [13]. In addition, lumbar traction does not improve spinal mobility. Some studies have reported that lumbar traction reduces the compression force on the intervertebral disc, reduces nerve root compression by expanding the intervertebral foramen, and helps the intervertebral disc return to its original position in the spinal ligament by generating tension [14]. Previous meta-analyses have confirmed that mechanical traction in the supine position can relieve short-term pain in patients with radiculopathy. Radical lesions include lumbar disc degeneration or hernia, degenerative arthritis, lumbar spinal stenosis, space-occupying lesions, and inflammatory lesions, which are distinguished from lumbar disc herniation. Previous meta-analyses have pointed out that mechanical traction and other noninvasive treatments could only improve symptoms in the short term [2]. However, there was heterogeneity among the literatures included in the analysis, especially regarding long-term treatment effects, the source of heterogeneity was not elucidated, and the confidence of the results was low. The study was limited to the effects of mechanical traction on lumbar pain and function and did not identify changes in ODI and Schober's test. That being said, it is necessary to further conduct a meta-analysis to explore the clinical effect of mechanical traction on patients with LDH. This analysis contributed significantly in understanding the basis for clinical diagnosis and provided novel insights on the relationship between mechanical traction and LDH.

## 2. Materials and Methods

### 2.1. Literature Download

Literature search was conducted in PubMed, Medline, Embase, CENTRAL, and CNKI databases. The main search terms were low back and leg pain or lumbar disc or lumbar disc herniation and traction or mechanical traction or physiotherapy or decompression. There were no restrictions on the language and publication time of the literature. The cut-off timeline for the literature search was set at April 23, 2022.

### 2.2. Literature Screening

Inclusion criteria are as follows: (1) the subjects were patients with lumbar disc herniation; (2) the study design included an experimental group and control group; (3) the experimental group received traction therapy combined with routine physical therapy, and the control group received routine physical therapy without traction; (4) provide efficacy evaluation before and after treatment, including visual analog scale (VAS), Oswestry disability index (ODI), and Schober test; and (5) randomized controlled study.

Exclusion criteria are as follows: (1) repeated reports; (2) the baseline data of the experimental group and the control group were unbalanced, with a statistical difference; (3) the experimental group or control group tried to apply intervention measures other than physical therapy; (4) the literature data is missing and cannot be supplemented by contacting the literature author.

### 2.3. Data Extraction

Two researchers jointly extracted the author, title, publication time, the number of researchers, efficacy evaluation results before and after treatment, etc. For the data that cannot be obtained in the literatures, researchers were responsible reaching out to the author for personal retrieval. If two researchers disagree on the data, an agreement was reached through discussion.

### 2.4. Literature Quality Evaluation

In this paper, two researchers used the Jadad scale, including the generation method of random sequence, the method of randomized hiding, the use of the blind method, and withdrawal rules, to evaluate the quality of the included studies. On the Jadad scale, 1 to 3 points are low quality, and 4 to 7 points are high quality.

### 2.5. Heterogeneity Test and Publication Bias Test

The Chi-square test was used for the heterogeneity test. When *I*^2^ corrected by degrees of freedom was more than 50% or *P* < 0.1, it was considered that there was heterogeneity among published literatures, and a random effect model was used. Subgroup analysis and sensitivity analysis were used to explore the causes of heterogeneity. When the *I*^2^ corrected by degrees of freedom is ≤50% and *P* ≥ 0.1, it was considered that there was no heterogeneity among the published literatures, and the fixed effect model was used. A funnel plot was used for the publication bias test.

### 2.6. Statistical Method

This study used Cochrane software RevMan5.3 to statistically analyze data. The variables included in this study are continuous variables. Mean difference (MD) and 95% confidence interval (CI) were used to describe the combined effect statistically. MD and 95% CI were calculated using the inverse variance statistical method. Bilateral *P* < 0.05 indicated statistically significant.

## 3. Results

### 3.1. Characteristics of Included Literature

A total of 1436 literatures were retrieved as described above. Screening through all literatures with defined criteria, there were 1430 literatures excluded and a total of 6 literatures included in this meta-analysis [15–20]. The working flow for screening is summarized in Figure 1. Further, the basic information of each literature and the in-detailed Jadad score are included in Table 1.

### 3.2. Comparison of VAS between Mechanical Traction and Conventional Physical Therapy

A total of 6 literatures involved the comparison of VAS of low back and leg pain after mechanical traction and conventional physical therapy. There were 239 patients in total with lumbar disc herniation, among whom, 123 cases in the mechanical traction group and 116 cases in conventional physical therapy. Heterogeneity test showed that there was no heterogeneity among the studies (Chi^2^ = 6.62, *P* = 0.25, and *I*^2^ = 24%). The combined analysis suggested that the VAS of patients in the mechanical traction group was lower than that in a routine physical therapy group with MD = −1.39 (95% CI (-1.81, -0.98)), and the difference was statistically significant (*Z* = 6.56, *P* < 0.00001). On top of that, as shown in the funnel diagram (Figure 2), scattered points were distributed in the confidence interval and were generally symmetrical. No publication bias was indicated in the study as shown in Figure 3.

### 3.3. Comparison of ODI between Mechanical Traction and Conventional Physical Therapy

Through screening, we identified 5 literatures which introduced a comparison of ODI after mechanical traction ad conventional physical therapy. Within the 5 literatures, there were total of 222 patients with lumbar disc herniation with 115 cases in the mechanical traction group and 107 cases in conventional physical therapy. The heterogeneity test showed that there was no heterogeneity among the studies (Chi^2^ = 6.27, *P* = 0.18, and *I*^2^ = 36%). Further analysis showed that the ODI of patients in the mechanical traction group was lower than that in a routine physical therapy group (MD = −6.34 95%, CI (-10.28, -2.39)), and the difference was statistically significant (*Z* = 3.15, *P* = 0.002). The funnel chart showed a roughly symmetrical distribution of the scatter points within the confidence interval (Figure 4). No publication bias was observed while conducting analysis (Figure 5).

### 3.4. Comparison between Mechanical Traction and Conventional Physical Therapy Schober Test

During the investigation of Schober test after mechanical traction and conventional physical therapy, there were 200 patients with lumbar disc herniation with 101 cases in the mechanical traction group and 99 cases in conventional physical therapy investigated in 5 screen literatures. The heterogeneity test showed no heterogeneity among the studies (Chi^2^ = 1.61, *P* = 0.66, and *I*^2^ = 0%). The combined analysis results showed that the Schober test score of patients in the mechanical traction group was lower than that in the conventional physical therapy group, MD = −0.40 (95% CI (-1.07, 0.28)), and the difference was not statistically significant (*Z* = 1.16, *P* = 0.25). Similar to other test, in Figure 6, the funnel chart showed that the scattered points were distributed semisymmetrical within the confidence interval. The publication bias screening showed no significant stand-out bias (Figure 7).

## 4. Discussion

The clinical efficacy of lumbar traction has been controversial, including in terms of long-term and short-term efficacy. We confirmed the short-term efficacy of limited lumbar traction through a meta-analysis. As published previously, mechanical traction could alleviate low back pain, reduce ODI, and improve symptoms in patients with lumbar disc herniation. Through our analysis, lumbar traction takes effects in two major ways. First of all, the vertebral bodies are separated through traction, which contributed to reduce the compressive force and further reduce the compression on the nerve root. The other way is to strengthen the role of the spinal ligaments and help the intervertebral disc reset. It has also been noted that lumbar traction is thought to alter disc size [2]. However, there is no evidence supporting such conclusion, and no theoretical basis was proposed.

We reviewed the literature included in the analysis. Bilgilisoy et al. [15] compared the effects of supine traction, prone traction, and conventional physical therapy on ODI, pain, and activity in patients with a lumbar disc. They suggested that mechanical traction can improve ODI and reduce pain, but it has no significant effect on activity. The study [15] also pointed out that mechanical traction in a prone position was better than in a supine position. In other studies, such as Demirel et al. [18] compared the efficacy of traction decompression with conventional physical therapy. From which, both treatments could reduce the pain symptoms of patients with lumbar disc herniation and promote the functional recovery of patients. This study [18] suggested traction decompression as an auxiliary physical therapy method for lumbar disc herniation. Isner-Horobeti et al. [19] further compared the efficacy of high-intensity and low-intensity lumbar traction in treating acute sciatica secondary to intervertebral disc herniation. Both high-intensity and low-intensity traction could reduce nerve root pain and improve patients' dysfunction and psychological state. The curative effect of high-intensity traction was better than that of low-intensity traction. The impact of mechanical traction had nothing to do with the initial amount of drug treatment, and the treatment effect could be maintained for at least 2 weeks. Moustafa and Diab [16] studied the effect of mechanical traction and physical therapy on unilateral lumbosacral radiculopathy caused by L5-S1 disc herniation. After 10 weeks of treatment, the traction group was better than the control group in ODI, low back and leg pain, modified Schober test, and intervertebral movement. At 6 months of follow-up, the difference between the traction group and the control group in the above variables was still statistically significant. However, the modified Schober test results of Moustafa and Diab [16] were inconsistent with our meta-analysis results. Other studies have also suggested that lumbar traction cannot improve spinal mobility [21, 22], which might be related to the strict restriction of the research object, meaning the inclusion of only patients with lumbar lordosis angle less than 39° might lead to more significant results. They also suggested a long-term effect was observed in 6-month follow-ups, which is controversial to other previous studies indicating that the curative effect of lumbar traction could only be reflected in the short term [2]. Ozturk et al. [20] studied the effect of continuous lumbar traction on the clinical and imaging manifestations of patients with lumbar disc herniation. The traction group was treated with physical therapy combined with continuous lumbar traction while the control group only received physical therapy. During Ozturk et al.'s study, patients with higher protrusion responded better to traction. Lumbar traction can not only effectively improve the clinical manifestations of patients with lumbar disc herniation but also reduce the degree of lumbar disc herniation. Prasad et al. [17] also concluded that intermittent traction combined with physical therapy could improve the clinical symptoms and function of lumbar disc herniation and improve the life treatment of patients. Intermittent traction could significantly reduce the need for surgery.

With all the strict analysis in this study, there are some limitations. The literature sizes and case sizes were limited by the strict criteria applied. In addition, sham traction controls and blank controls were included in the included studies, which may have had some impact on the results. Larger randomized controlled trials are still needed to confirm the therapeutic effect of mechanical traction on lumbar disc herniation.

Mechanical traction is a way of physical therapy which can effectively reduce the low back and leg pain and improve ODI in patients with lumbar disc herniation. Still, it has no significant effect on the spine's range of motion. The therapeutic effect of mechanical traction is significantly better than that of conventional physical therapy. Lumbar traction can be combined with other conventional physical therapy.

## Figures and Tables

**Figure 1:** Document screening flow chart.

**Figure 2:** Forest diagram of VAS comparison between mechanical traction and conventional physical therapy groups.

**Figure 3:** Funnel diagram of VAS comparison between mechanical traction and routine physical therapy groups. MD means mean difference; SE stands for standard error.

**Figure 4:** Forest diagram of ODI comparison between mechanical traction and conventional physical therapy.

**Figure 5:** Funnel diagram of ODI comparison between mechanical traction and conventional physical therapy. MD means mean difference; SE stands for standard error.

**Figure 6:** Forest diagram of comparison between mechanical traction and conventional physical therapy Schober test.

**Figure 7:** Funnel diagram of comparison between mechanical traction and conventional physical therapy Schober test. MD means mean difference; SE stands for standard error.

**Table 1:** Literature characteristics and Jadad score were included.

Author	Year	Study type	Study group	Control group	Frequency (times/week)	Traction	Jadad
Bilgilisoy et al. [15]	2018	RCT	*n* = 39 Age: 45.1 ± 11.2	*n* = 40 Age: 45.1 ± 11.2	Not mentioned	50%BW	4
Demirel et al. [18]	2017	RCT	*n* = 10 Age: 50.1 ± 11.8	*n* = 10 Age: 41.3 ± 12.8	Not mentioned	50%BW+5 pounds	5
Isner-Horobeti et al. [19]	2016	RCT	*n* = 8 Age: 33 ± 11	*n* = 9 Age: 33 ± 8	5	50%BW	4
Moustafa and Diab [16]	2013	RCT	*n* = 30 Age: 43.2 ± 2.4	*n* = 28 Age: 43.2 ± 1.7	3	Not mentioned	5
Ozturk et al. [20]	2006	RCT	*n* = 24 (14 men, 10 women) Age: 40.2 ± 11.4	*n* = 22 (8 men, 14 women) Age: 52.7 ± 8.8	5	50%BW	5
Prasad et al. [17]	2012	RCT	*n* = 12 Age: 36.55 ± 5.13	*n* = 7 Age: 34.46 ± 5.71	3	Not mentioned	5

RCT: randomized controlled trial.

## Data Availability

The data used to support the findings of this study are included within the article.
